# circZNF91 Promotes the Malignant Phenotype of Chronic Lymphocytic Leukemia Cells by Targeting the miR-1283/WEE1 Axis

**DOI:** 10.1155/2022/2855394

**Published:** 2022-05-05

**Authors:** Shaoting Li, Jing Chen, Ying Fan, Xiaoli Xu, Minjian Xiong, Yonglei Qi, Wenlin Wu, Ying Zhao

**Affiliations:** ^1^Department of Pharmacy, The Fifth Hospital of Wuhan, Hubei 430050, China; ^2^Department of General Medicine, Erqiao Street Community Health Service Center Affiliate of the Fifth Hospital of Wuhan, Wuhan, Hubei 430050, China; ^3^Department of Cardiology, The Fifth Hospital of Wuhan, Wuhan, Hubei 430050, China; ^4^Department of Hematology, The First People's Hospital of Foshan, Foshan, Guangdong 528000, China; ^5^Department of Internal Medicine, Parrot Street Community Health Service Center Affiliate of the Fifth Hospital of Wuhan, Wuhan, Hubei 430050, China

## Abstract

**Background:**

Circular RNAs (circRNAs) are frequently dysregulated in cancers and are implicated in tumorigenesis and tumor progression. In this study, we investigated the role of circZNF91 in regulating the malignant phenotype of chronic lymphocytic leukemia (CLL) cells and the underlying molecular mechanism.

**Material:**

/

**Methods:**

The expression of circZNF91 was determined by reverse transcription-quantitative polymerase chain reaction (RT-qPCR). The binding sequences between circZNF91/miR-1283 and miR-1283/WEE1 were predicted by the bioinformatic database. The functional interactions were confirmed by the dual-luciferase reporter, RT-qPCR, and Western blot assays. The functional roles of the circZNF91/miR-1283/WEE1 axis in CLL progression were examined by cell proliferation, apoptosis, and EdU incorporation assays.

**Results:**

circZNF91 was upregulated in CLL samples. Silencing circZNF91 attenuated CLL cell proliferation and induced apoptosis and cell cycle arrest. circZNF91 could sponge miR-1283 to suppress its activity, which in turn upregulated WEE1 expression. Silencing circ-TTBK2 reduced WEE1 expression, while the inhibitor of miR-1283 enhanced WEE1 expression. The miR-1283/WEE1 axis mediated the effects of circZNF91 on cell proliferation and apoptosis, as well as induced cell cycle regulation.

**Conclusions:**

The circZNF91/miR-1283/WEE1 axis is engaged in the pathological phenotypes of CLL cells, which could serve as potential targets for future therapy development.

## 1. Introduction

Chronic lymphocytic leukemia (CLL) is a common type of cancer in the blood and bone marrow, and the underlying pathogenesis has not been fully understood. Circular RNAs (circRNAs) are a class of noncoding RNAs implicated in many diseases and pathological conditions, including cancers [1]. For example, in oral squamous cell carcinoma, hsa_circRNA_100290 is overexpressed and could interact with miR-378a to regulate the progression of squamous cell carcinoma through the miR-136-5p/RAP2C axis [2]. In addition, circZNF91 is another circRNA that is frequently aberrantly expressed and functions as a sponge to target downstream microRNAs in many cancers [3]. However, the potential role and mechanism of circZNF91 in CLL remain unknown.

The biological roles of circRNAs are frequently associated with target microRNAs (miRNAs) [4]. miRNAs are linear noncoding RNAs, while circRNAs have closed-loop structures, which make circRNAs more stable than miRNAs [5, 6]. When interacting with miRNAs, circRNAs act as specific “sponges” or “reservoirs” for miRNAs, by which they competitively bind to miRNAs and interfere with the pairing of miRNAs and downstream target mRNAs [7]. For example, the knockdown of circ-TTBK2 inhibits glioma progression by sponging miR-1283 [8]. However, the expression pattern and role of miR-1283 in the context of CLL remain to be investigated.

In this study, we examined the expression pattern and functional role of circZNF91 in CLL. We further identified the target miRNA and downstream mRNA *via* bioinformatic database prediction, which were confirmed by dual-luciferase reporter assay and RT-qPCR. Furthermore, their functional interactions were examined by cellular assays, including cell proliferation, apoptosis, and EdU staining assays. Our data showed that circZNF91 is upregulated in CLL and silencing circZNF91 attenuated CLL cell proliferation and induced apoptosis and cell cycle arrest. We further showed that the miR-1283/WEE1 axis mediates the functional effects of circZNF91 on CLL cells. Our study suggests that the circZNF91/miR-1283/WEE1 axis may be engaged in the progression of CLL and understanding the dysregulation of circZNF91 could provide insights into novel therapy development of CLL.

## 2. Materials and Methods

### 2.1. Reagents

Roswell Park Memorial Institute- (RPMI-) 1640 medium and Dulbecco's modified Eagle's medium (DMEM) were purchased from Invitrogen (Carlsbad, CA, USA). Small interfering RNA (siRNA) targeting circZNF91 (shcirc#1, sh-circ#2, and sh-circ#3) and corresponding negative control (sh-NC), miR-1283 mimic or inhibitor (miR-296-5p, or anti-miR-296-5p), and corresponding negative controls (miR-NC or anti-NC) were purchased from Genechem (Shanghai, China). Oligonucleotides (working concentration 50 nM) or vectors (working concentration 2 *μ*g) were purchased from Integrated DNA Technologies (Coralville, IA, USA). Lipofectamine™ 3000 and other transfection reagents were obtained from Invitrogen. Primary antibodies and horseradish peroxidase-linked secondary antibody were obtained from Abcam (Cambridge, MA, USA).

### 2.2. Patient Sample Collection

A total number of 45 patients who were diagnosed with CLL were enrolled in this study. The blood samples of the 45 individuals and 20 healthy controls were collected at the department of hematology, The First People's Hospital of Foshan, between June 2019 and July 2020. The samples were immediately frozen in liquid nitrogen and then stored in a −80°C deep freezer. All enrolled individuals signed informed consent.

Inclusion criteria are as follows: subjects who were able to provide written informed consent to participate in the study on a voluntary basis, subjects who had no other concurrent malignant tumors, and subjects who had no blood-related diseases and infectious diseases observed. Exclusion criteria are as follows: subjects who were undergoing chemotherapy, subjects who had fatal diseases, and subjects diagnosed with other types of tumors.

### 2.3. Cell Culture and Transfection

MEC-1 cells were cultured with RPMI-1640 medium, and the HG-3 cells were cultured in DMEM medium, supplemented with 10% FBS and 1% penicillin/streptomycin (Invitrogen). To investigate the role of circZNF91, MEC-1 cells and HG-3 cells were transfected with 100 nM siRNA targeting circZNF91. For miRNA, cells were transfected with 50 nM of mimics and controls or inhibitors. Transfection was performed with Lipofectamine™ Stem Reagent (STEM00001, Invitrogen). In a 6-well plate, 60% confluent cells were transfected with 50 nM of a microRNA mimic/inhibitor, 2 *μ*g of plasmid, or 100 nM siRNA, according to the manufacturer's instructions. Transfected cells were subjected to subsequent analysis 48 h posttransfection.

### 2.4. Dual-Luciferase Reporter Assay

The CircInteractome database was used to predict the binding sequence between target miRNAs of circZNF91. The mRNA target of miR-1283 was analyzed by TargetScan (http://www.targetscan.org/). To confirm predicted binding, the sequence containing the wild-type (WT) binding site and the sequence with the mutated (MUT) binding site were cloned into the pmirGLO vector expressing firefly luciferase, respectively (Promega, E1330). The reporter plasmid and Renilla luciferase (hRlucneo) control plasmid were cotransfected into cells with either miR-1283 mimic or miR-NC in a 12-well plate (1 × 10^5^ cells/well). 48 h posttransfection, luciferase activities were measured using a dual-luciferase reporter assay kit (Promega) on a luminescence microplate reader.

### 2.5. Western Blotting

Proteins from the CLL cells were extracted by lysis buffer (Beyotime, Nanjing, China). After examining the concentration of protein with the BCA kit, denatured samples were separated by sodium dodecyl sulfate-polyacrylamide gel electrophoresis (SDS-PAGE) and then transferred onto the PVDF membrane. After blocking with 5% skimmed milk for 1 h, the membrane was then incubated with primary antibodies: cleaved caspase 3, CCND1, ki67, and GAPDH (1 : 1000 dilution) at 4°C. The membrane was washed 3 times with TBST buffer and was further incubated with HRP-linked secondary antibody (1 : 3000 dilution) at room temperature for 1 h. Then, the membrane was washed 4 times with TBST buffer, and the bands were visualized using an enhanced chemiluminescence kit (Santa Cruz) and photographed on a gel imager system (Bio-Rad, Hercules, CA, United States).

### 2.6. Reverse Transcription-Quantitative Polymerase Chain Reaction (RT-qPCR)

Total RNA from CLL tissues and cells was extracted using an RNA extraction kit (Invitrogen, CA, USA). 5 *μ*g of total RNA was used for reverse-transcription into cDNA using the PrimeScript™ RT Reagent Kit (TaKaRa Biotechnology RR037B, Otsu, Japan). The resultant cDNA was diluted and analyzed in a 7500 Real-Time PCR System (Applied Biosystems/Life Technologies, Carlsbad, CA, USA) using SYBR Green RT-qPCR SuperMix UDG Reagents (Invitrogen, CA, USA). The following PCR cycling conditions were used: 95°C for 2 min, 40 cycles of 95°C of 30 sec, 60°C for 30 sec, and 72°C for 60 sec, with signal detection at the end of each cycle. Finally, the 2^–∆∆*Ct*^ method was used to analyze the relative expression level. GAPDH and U6 were used as the internal reference genes. All primer sequences were synthesized and purchased from Sangon Biotechnology Ltd. (Shanghai, China), which are listed in Table 1.

### 2.7. Cell Proliferation Assay

After 48 h of transfection, cells were seeded in a 96-well plate at a density of 1500 cells/well and cultured in a humidified cell culture incubator for 0, 24, 48, and 72 h. Subsequently, 10 *μ*L of CCK-8 working solution (Solarbio, CA1210, Beijing, China) was added to the cell culture at the indicated time point and incubated for 1 h. The light absorption value (OD value) in each condition was captured at 450 nm wavelength on Cytation 5 Cell Imaging Multi-Mode Reader.

### 2.8. Edu Incorporation Assay

Edu incorporation assay was performed using the EdU Cell Proliferation Assay Kit (**#** 1329, Click Chemistry Tools). The prewarmed 2x EdU solution was added in an equal volume into the cell culture medium for 2 h incubation. Cells were washed twice with PBS, followed by fixation with 100 *μ*L of 3.7% formaldehyde in PBS for 15 min at room temperature. After the removal of the fixative solution, cells were washed twice with 100 *μ*L of PBS with 3% BSA. Then, 100 *μ*L of 0.5% Triton® X-100 in PBS was added to each well for 20 min incubation. After the removal of the solution, 1 × Click-iT® reaction cocktail was prepared based on the manufacturer's instructions and added to cells for 30 min. The staining cocktail was removed, and cells were washed twice with 100 *μ*L of PBS with 3% BSA. Cells were counterstained by 500 nM DAPI in PBS, and the images were captured under a Leica AM6000 microscope.

### 2.9. Cell Cycle Analysis

Cells were harvested in single-cell suspension in buffer (PBS + 2% FBS). Cells were washed and resuspended at the density of 1 × 10^6^ cells/mL. 5 mL of cold 70% ethanol was added dropwise into the cell suspension in a 15 mL polypropylene tube and incubated at −20°C for 16 h prior to PI staining. Cells were centrifuged at 1000 × g for 5 min, and the pellet was washed twice in PBS. Propidium iodide was added at a concentration of 50 mg/mL for 4 h staining and analyzed by flow cytometry.

### 2.10. Apoptosis Assay

Apoptosis assay was performed by the FITC Annexin V Apoptosis Detection Kit (BD Biosciences, PharMingen, San Jose, CA, USA) according to the manufacturer's instructions. Cells were seeded in a 6-well plate at a density of 1 × 10^6^ cells/well and transfected with indicated molecules. After 48 h of transfection, 5 *μ*L of Annexin V-FITC and 5 *μ*L of PI were added to the 1000 *μ*L of cell resuspension with 5 × 10^5^ cells and incubated for 30 min in the dark. Stained cells were washed twice with PBS and resuspended in 400 *μ*L of PBS. The percentage of apoptotic cells was detected by a BD FACSCanto™ II Flow Cytometer (BD Biosciences).

### 2.11. RNA Immunoprecipitation

RNA immunoprecipitation (RIP) assays were performed using the EZMagna RIP kit (Millipore). The lysate was incubated with Pierce™ Protein A/G Magnetic Beads (Thermo Fisher Scientific, 88803) conjugated with a rabbit anti-Ago2 (Abcam, ab32381) antibody or with a negative control normal rabbit anti-IgG (Abcam, ab188776). The mixture was incubated at 4°C with shaking overnight. Magnetic beads were precipitated using a magnetic bar, and the precipitated samples were washed three times with NT2 buffer. The eluted samples were purified with TRIzol reagent (Invitrogen, 15596026) and analyzed by RT-qPCR.

### 2.12. RNA Pull-Down Assay

Cell lysates were collected by IP lysis buffer (Beyotime, P0013) and were incubated biotinylated miR-1283 oligo and miR-NC oligos. 10% of the lysate was saved as the input. The mixture was further incubated with M-280 streptavidin magnetic beads (Sigma-Aldrich, 11205D) at 4°C shaking overnight. A magnetic bar was used to pull down the magnetic beads and associated nucleic acids. After 4 washes with high salt wash buffer, the input and the elutes from the pull down were purified with TRIzol reagent and the relative level of circZNF91 was analyzed by RT-qPCR.

### 2.13. Statistical Analysis

All data were analyzed by GraphPad Prism 8 software. The association between circZNF91 expression and the clinic pathological parameters was evaluated with the chi-square analysis. The statistical difference between the two groups was examined using unpaired Student's *t*-tests. Comparisons among multiple groups were analyzed using a one-way analysis of variance (ANOVA) with Tukey's post hoc test. The Kaplan-Meier curve and log-rank test were used to compare the cumulative survival rates. Data were reported as the mean ± standard deviation (SD). ^∗^*P* < 0.05, ^∗∗^*P* < 0.01, and ^∗∗∗^*P* < 0.001; ^#^*P* < 0.05, ^##^*P* < 0.01, and ^###^*P* < 0.001.

## 3. Results

### 3.1. circZNF91 Is Upregulated in CLL Specimens and Cells

Initially, we compared the expression level of circZNF91 in the peripheral blood of normal individuals (*n* = 20) and CLL patients (*n* = 45). circZNF91 was significantly upregulated in the CLL specimens (Figure 1(a)). Similarly, compared with peripheral blood mononuclear cells (PBMCs), circZNF91 was upregulated in CLL cell lines, such as MEC-1 and HG-3 (Figure 1(b)). We next examined the area under the curve (AUC) of circZNF91 with the ROC curve. As shown in Figure 1(c), the AUC is larger than 0.8, which indicates the reliability of circZNF91 as the diagnostic biomarker. The CLL patients were divided into patients with high circZNF91 expression (*n* = 22) and low expression (*n* = 23) based on the median expression value of circZNF91. Kaplan-Meier analysis showed that high circZNF91 expression was associated with a worse survival rate in CLL patients (Figure 1(d)).

### 3.2. Knockdown of circZNF91 Inhibits CLL Cell Growth and Induces Apoptosis as well as Cell Cycle Arrest

To verify the biological function of circZNF91 in CLL cells, we silenced circZNF91 expression in MEC-1 and HG-3 cells using siRNA. The expression of circZNF91 was significantly decreased in MEC-1 and HG-3 cells transfected with three different siRNAs targeting circZNF91, with si-circZNF91#1 showing the best knockdown efficacy (Figure 2(a)). Thus, si-circZNF91#1 was used in the following experiments. CCK-8 proliferation assay demonstrated that compared with that of the si-NC group, the knockdown of circZNF91 inhibited the proliferative ability of MEC-1 and HG-3 cells (Figure 2(b)). EdU incorporation assay further showed that silencing circZNF91 significantly suppressed DNA synthesis (Figure 2(c)). The percentage of apoptotic events was significantly increased upon circZNF91 silencing (Figure 2(d)). Furthermore, circZNF91 knockdown increased the percentage of cells in the G0/G1 phase, which indicates a G1/S arrest in the cell cycle (Figure 2(e)). These results were consistent with the downregulation of Ki67 and cyclin D1 upon the knockdown of circZNF91, which are markers for cell proliferation and cell cycle progression, respectively, while the apoptotic marker cleaved caspase-3 was increased (Figure 2(f)). These data suggest that circZNF91 is required for the proliferation and survival of CLL cells.

### 3.3. circZNF91 Serves as a Sponge of miR-1283

Next, we investigated the intracellular localization of circZNF91 in MEC-1 and HG-3 cells. circZNF91 was predominantly detected in the cytoplasmic fraction of cells (Figure 3(a)). We next used the CircInteractome database to predict the potential miRNA targets of circZNF91. It was observed that miR-1283 contained a potential biding site for circZNF91 (Figure 3(b)). To validate the functional interaction between miR-1283 and circZNF91, we performed a dual-luciferase assay using WT and MUT reporters containing a mutated binding site in the presence of miR-1283 mimic. The miR-1283 mimic can significantly increase the cellular level of miR-1283 (Figure 3(c)). The presence of miR-1283 mimic could significantly suppress the luciferase activity in the WT reporter, but no effect was observed in the MUT reporter (Figure 3(d)). RNA pull-down assay using biotin-labeled oligos further showed that the biotin-miR-1283 probe could significantly enrich circZNF91 (Figure 3(e)) and RIP assay using anti-Ago2 antibody showed that Ago-2 protein could interact with both miR-1283 and circZNF91 (Figure 3(f)). These results strongly suggest the direct interaction between miR-1283 and circZNF9. Additionally, the expression of miR-1283 was reduced in the blood samples of CLL patients as compared to healthy controls (Figure 3(g)). Spearman correlation coefficient analysis indicated the negative correlation between the expression of circZNF91 and the expression of miR-1283 in CLL patients (Figure 3(h)). Together, these results suggest that circZNF91 could act as a sponge of miR-1283 in CLL cells.

### 3.4. Overexpression of miR-1283 Suppresses Proliferation and Induces Apoptosis as well as G1/S Arrest

To further investigate the role of miR-1283 in CLL, we transfected MEC-1 and HG-3 cells with miR-1283 mimic to overexpress miR-1283. miR-1283 overexpression suppressed cell proliferation in MEC-1 and HG-3 cells (Figure 4(a)), as well as the incorporation of EdU in DNA synthesis (Figure 4(b)). miR-1283 mimic also significantly promoted apoptosis (Figure 4(c)) and induced G1/S arrest in both cell lines (Figure 4(d)). These results were consistent with the downregulation of Ki67 and cyclin D1 and the increased level of apoptotic marker cleaved caspase-3 upon miR-1283 overexpression (Figure 2(e)). These data suggest that miR-1283 overexpression recapitulates the effect of circZNF91 silencing.

### 3.5. WEE1 Is a Downstream Target of miR-1283

We next searched for the downstream target of miR-1283. WEE1 mRNA was found to contain a potential binding site for miR-1283 *via* bioinformatics analysis. The potential binding site of miR-1283 in the 3′-UTR of WEE1 is shown in Figure 5(a). Dual-luciferase reporter experiment revealed that miR-1283 mimic could inhibit the luciferase activity of the WEE1-WT reporter, while no effects were observed in the mutated reporter (Figure 5(a)). We also applied miR-1283 inhibitor, which can suppress the level of miR-1283 (Figure 5(b)). We transfected MEC-1 and HG-3 cells with miR-1283 mimic, inhibitor, and corresponding controls and performed a Western blot assay to examine the protein level of WEE1. miR-1283 overexpression suppressed WEE1 expression while the miR-1283 inhibitor increased the WEE1 level (Figure 5(c)). These data suggest that WEE1 is a target negatively regulated by miR-1283. In the published GSE222529 dataset, WEE1 is highly expressed in CLL patients (Figure 5(d)). RT-qPCR analysis in the blood samples of CLL patients and healthy controls in our study also confirmed the upregulation of WEE1 in CLL patients (Figure 5(e)). We further measured the correlation between miR-1283 and WEE1, circZNF91, and WEE1 *via* Spearman's correlation analysis. We observed a negative correlation between miR-1283 and WEE1 expression levels and a positive correlation between circZNF91 and WEE1 expression (Figures 5(f) and 5(g)).

### 3.6. miR-1283/WEE1 Mediates the Effect of circZNF91

To further explore the functional interactions among circZNF91, miR-1283, and WEE1 in CLL, cells were silenced by circZNF91 siRNA alone or cotransfected with the miR-1283 inhibitor or WEE1 expression vector. Western blot revealed that both the miR-1283 inhibitor and WEE1 overexpression rescued the WEE1 expression level after circZNF91 silencing (Figure 6(a)). CCK-8 proliferation assay demonstrated that the miR-1283 inhibitor or WEE1 overexpression could partially rescue the proliferation after circZNF91 silencing (Figure 6(b)), as well as the EdU incorporation for DNA synthesis (Figure 6(c)). These effects were accompanied by a reduced level of apoptosis and attenuated G1/S phase arrest (Figures 6(d) and 6(e)). Meanwhile, both the miR-1283 inhibitor and WEE1 overexpression suppressed the level of cleaved caspase-3 and increased the level of Ki67 and cyclin D (Figure 6(f)). Together, these data showed that miR-1283/WEE1 mediated the effect of circZNF91.

## 4. Discussion

circRNAs are widely expressed in many species, and their aberrant expression is associated with the pathological condition such as cancer progression [9, 10]. They are characterized by stability (resistance to enzymes, such as RNase R due to the circular structure) [11, 12], high level of conservation (highly conserved between humans and other species) [13], and specificity (expressions are specifically induced by certain conditions) [14–16].

In our study, we demonstrated the upregulation of circZNF91 in the blood sample of CLL cancer patients. circZNF91 was mainly located in the cytoplasm of the CLL cancer cell line (MEC-1 and HG-3), having high expression cis associated with a poorer prognosis in CLL patients. This suggests that circZNF91 may serve as a prognostic marker. We further showed that knockdown of circZNF91 suppressed the proliferation of CLL cells and induced apoptosis and G1/S arrest, indicating that circZNF91 is indispensable for the sustained proliferation of CLL cells. Although we did not examine the mechanism by which the G1/S arrest is induced upon circZNF91 silencing, we speculate that the downregulation of cyclin D1 (CCND1) may account for the blockade of cells in the G1/S checkpoint. However, a detailed investigation of the interplay between circZNF91 and cyclin D1 expression could provide novel insights into how circZNF91 regulates cell cycle progression.

Our study further clarified that circZNF91 acts as a sponge for miR-1283 and negatively regulates the expression of miR-1283. Their interaction was validated by dual-luciferase reporter assay and RNA pull-down assay. Importantly, the overexpression of miR-1283 using miR-1283 mimic recapitulates the biological effects of circZNF91 knockdown, suggesting that miR-1283 is a downstream mediator of circZNF91.

Further, we revealed that miR-1283 binds to and negatively regulates the mRNA of WEE1. WEE1 is a nuclear kinase that is upregulated in many cancers and is proposed as a target for anticancer therapy [17, 18]. It is capable of regulating cell cycle progression [17, 19]. In addition, WEE1 expression has been considered as a novel prognostic marker associated with poor outcomes [20–22]. Our study showed that circZNF91 suppresses the activity of miR-1283, which releases its inhibition of WEE1 expression. WEE1 overexpression could rescue the effect of circZNF91 silencing on cell proliferation, apoptosis, and cell cycle arrest. Interestingly, a WEE1 chemical inhibitor MK-1775/AZD1775 could partially prevent metastasis through interfering S phase and G2/M phase in the cell cycle [23]. However, the mechanism by which WEE1 regulates cell cycle progression in CLL remains to be elucidated.

Notably, there are several questions remaining to be answered regarding the circZNF91/miR-1283/WEE1 axis in the regulation of CLL progression. First, how circZNF91 becomes dysregulated in CLL is unclear. Second, whether WEE1 is the only target that mediates the downstream effect needs to be clarified. Additionally, the functional role of circZNF91 in CLL needs to be investigated in the animal model.

## 5. Conclusion

In this study, we demonstrated the upregulation of circZNF91 in CLL patients and cell lines and its critical role in supporting CLL progression. circZNF91 interacted with miR-1283 and negatively regulated miR-1283 expression. The sponging effect of circZNF91 on miR-1283 relieved its inhibition of WEE1 expression. The miR-1283 inhibitor or WEE1 overexpression could partially reverse the effects of circZNF91 knockdown in CLL cells. Therefore, our study revealed a novel functional role of the circZNF91/miR-1283/WEE1 axis in CLL progression.

## Figures and Tables

**Figure 1:** The level of circZNF91 in CLL patients. (a) The expression levels of circZNF91 in peripheral blood of normal individuals (*n* = 20) and CLL patients (*n*  = 45) were detected by RT-qPCR. (b) circZNF91 expression in PBMC (peripheral blood mononuclear cell) and CLL cell lines (MEC-1 and HG-3). (c) circZNF91 expression in peripheral blood of CLL patients was analyzed by the ROC curve. (d) The overall survival rates of CLL patients with low expression of circZNF91 (*n* = 23) and high expression of circZNF91 (*n* = 22) were evaluated by the Kaplan-Meier survival curve.

**Figure 2:** Knockdown of circZNF91 inhibits the proliferation of CLL cells and induces apoptosis and G1/S cell cycle arrest. (a) The knockdown efficiency of siRNAs targeting circZNF91 in MEC-1 and HG-3 (Si-NC and si-circZNF91#1, si-circZNF91#2, and si-circZNF91#3). (b) CCK proliferation assay at 0 h, 24 h, 48 h, and 72 h. (c) EdU incorporation assay in cells transfected with si-NC and si-circZNF91#1. (d) Apoptotic assay in cells transfected with si-NC and si-circZNF91#1. (e) Cell cycle analysis in cells transfected with si-NC and si-circZNF91#1. (f) The protein levels (Ki-67, cleaved caspase 3, and CCND1) in MEC-1 and HG-3 cells transfected with si-NC and si-circZNF91#1 were detected by Western blot.

**Figure 3:** cirZNF91 interacts with miR-1283 in CLL cells. (a) The subcellular localization of circZNF91 was detected in MEC-1 and HG-3 cells. The expression level of circZNF91 in the nucleus and cytoplasm was detected by RT-qPCR. (b) The binding site of circZNF91 and miR-1283 was predicted by CircInteractome. (c) miR-1283 expression level after the transfection with miR-1283 mimic or miR-NC. (d) A dual-luciferase assay using WT and MUT reporters, in the presence of miR-1283 mimic or miR-NC. (e) RNA pull-down assay using biotin-labeled miR-NC or miR-1283 probe. (f) The enrichment of miR-1283 and cirZNF91 in MEC-1 and HG-3 cells was detected by RIP (RNA immunoprecipitation) assay after incubation with anti-Ago2 or anti-IgG. (g) The expression level of miR-1283 in 20 normal subjects and 45 CLL patients was detected by RT-qPCR. (h) A negative correlation between the expression of circZNF91 and miR-1283 in CLL was detected by Spearman correlation coefficient analysis.

**Figure 4:** Overexpression of miR-1283 inhibits the proliferation of CLL cells and induces apoptosis and G1/S arrest. Cells were transfected with miR-NC and miR-1283-mimic. (a) CCK-8 proliferation assay, (b) EdU incorporation assay, (c) apoptosis assay, (d) cell cycle analysis, and (e) Western blot analysis of Ki-67 cleaved caspase 3 and CCND1 (cyclin D) were performed in cells (miR-NC and miR-1283).

**Figure 5:** miR-1283 targets WEE1. TargetScan was used to predict the binding site of miR-1283 between WEE1 mRNAs. A dual-luciferase assay was performed using WT and MUT reporters. (b) RT-qPCR was used to detect the expression of miR-1283 after the transfection with the miR-1283 inhibitor. (c) The protein level of WEE1 in MEC-1 and HG-3 cells of different groups (miR-NC, miR-1283, NC inhibitor, and miR-1283 inhibitor). (d) WEE1 expression in CLL patients and healthy controls was analyzed using the GSE222529 dataset. (e) The expression level of WEE1 in normal subjects (*n* = 20) and CLL patients (*n* = 45) was examined by RT-qPCR. (f) Negative correlation between miR-1283 and WEE1 expression in CLL by Spearman correlation coefficient. (g) Positive correlation between circZNF91 and WEE1 expression in CLL by Spearman correlation coefficient analysis.

**Figure 6:** The miR-1283/WEE1 axis mediates the effect of circZNF91. Cells were transfected with si-NC or si-circZNF91. In the si-circ-ZNF91 group, cells were further cotransfected with the miR-1283 inhibitor or WEE1 overexpression vector. (a) The expression levels of WEE1 protein in the above cells were detected by Western blot. (b) Cell proliferation, (c) EdU incorporation assay, (d) apoptosis assay, (e) cell cycle analysis, and (f) protein expression levels of Ki-67, cleaved caspase 3, and CCND1 were analyzed by Western blot.

**Table 1:** The list of prime sequences.

Name	Sequence
circZNF91 (divergent primer)	Forward: 5′-CTTTTC TGGGCCAAATCGG-3′ Reverse: 5′-ACGGG TACCGACGGGTC-3′
miR-1283	Forward: 5′-GGGAGAUCAGGUUCGGUCAGAG-3′ Reverse: 5′-CTGCCTGCATTC CTCTCAGA-3′
GAPDH	Forward: 5′-CGCGATGGAGAACCCAGAT-3′ Reverse: 5′-GGGCTTGTACCATAGATGAC-3′
U6:	Forward: 5′-ATCCGGCAGATGGCTGTTGAC-3′ Reverse: 5′-GGCCGGTACACCATTCCGATTC-3′
miR-1283 mimic	5′-UCUACAAAGGAAAGCGCUUUCU-3′
miR-NC	5′-UUCUCCGAACGUGUCACGUTT-3′
miR-1283 inhibitor	5′-AGAUGUUUCCUUUCGCGAAAGA-3′
Negative controls	5′-CAGUACUUUUGUGUAGUACAA-3′

## Data Availability

The data used to support the findings of this study are included within the article.
